This article has been retracted.

# Prevalence and associated factors of early initiation of breastfeeding among women delivered via Cesarean section in South Gondar zone hospitals Ethiopia, 2020

**DOI:** 10.1186/s40748-020-00121-3

**Published:** 2020-12-09

**Authors:** Bekalu Getnet, Alemu Degu, Fantahun Yenealem

**Affiliations:** 1 Department of Midwifery, College of Health Sciences, Debre Tabor University, P. Box: 272, Debre Tabor, Ethiopia; 2 Department of Midwifery, College of Medicine and Health Sciences, Bahir Dar University, Bahir Dar, Ethiopia

**Keywords:** Early initiation of breastfeeding, Cesarean delivery, Ethiopia

## Abstract

**Background:**

Early initiation of breastfeeding is putting the newborn to breast within one hour after birth. This study was aimed to assess prevalence of early initiation of breastfeeding and its associated factors among mothers who delivered by cesarean section in South Gondar Zone hospitals Northwest Ethiopia, 2020.

**Methods:**

An institutional based cross-sectional study was employed in South Gondar Zone hospitals from June 12 to July 03, 2020. A total of 356 cesarean delivered mothers were included. Data were collected using interviewer administered questionnaire and entered in to Epi Data version 4.2 and then exported to SPSS version 23.0. Logistic regression statistical analyses were used to identify factors associated with the outcome variables.

**Results:**

The prevalence of early initiation of breastfeeding among mothers who delivered by cesarean section was 51.9%. Mothers who had intended pregnancy [AOR = 2.69, 95% CI (1.34–5.38)], had professional guidance [AOR = 2.68, 95% CI (1.18–6.10)], had breastfeeding experience [AOR = 2.25, 95% CI (1.35–3.75)], and had four and above antenatal care visits [AOR = 2.20, 95% CI (1.24–3.91)] were positively associated with early initiation of breastfeeding among mothers who delivered by cesarean section.

**Conclusion:**

Type of pregnancy, professional guidance, had four or more antenatal care and breastfeeding experience were significantly associated with early initiation of breast feeding among mothers who delivered by cesarean section. Community based breastfeeding education and counseling to pregnant mothers and encouraging all mothers to follow recommended ANC visit is should be recommended.

## Introduction

Breastfeeding (BF) is the process of feeding the infant with the mother’s milk either pumped or expressed [1]. It also a key public health strategy to reduce infant, child, and maternal morbidity and mortality and helps to control health care costs [2].

Early breastfeeding initiation (EIBF) is described as breastfeeding of the newborn within one hour of birth and is the easiest, most cost-effective, and most successful intervention. It is one of the 10 steps of successful BF practice and one of the key indicators for assessing appropriate infant and young child feeding practices [3].

The importance of early initiation of breastfeeding could increase the likelihood of success in breastfeeding [4–6].

Delivery by cesarean section is an operational approach that substitutes the natural delivery process. Its rate has continued to rise over the last few decades, and further research has also shown that delivery by cesarean section is associated with non-initiation or delayed initiation of breastfeeding as well as with discontinuation of exclusive breastfeeding [7].

According to UNICEF’s recent survey, 78 million or 60 % of infants were not breastfed within the first hour of birth, results putting them at risk of illness and even death [8].

Neonatal hypothermia and infection are among the different causes of neonatal death due to delayed breastfeeding initiation (DIBF) [9].

In developing countries alone, an EIBF could save as many as 1.45 million lives each year by reducing deaths mainly due to diarrheal disorders and lower respiratory tract infections in children [10]; However, children also die from diarrheal disorders and low respiratory tract infections in the area due to DIBF [11].

In Ethiopia, making it 6th highest neonatal mortality in the world, and children are still dying in large numbers from preventable and treatable causes, like DIBF [12].

The prevalence of early initiation of breastfeeding increased from 48.8% in 2000 to 75.7% in 2016 in Ethiopia [13].

Cesarean Delivery (CD) is also one of the factors that may influence the initiation and continuation of breastfeeding, however findings are inconsistent and showed that CD had a detrimental effect on the mother’s ability to initiate and sustain breastfeeding [14, 15].

Other factors following the review of the literature have also shown that residence, maternal education, and occupation, maternal knowledge of the EIBF, breastfeeding experience, visit the ANC, number of visits to the ANC, EIBF support during the ANC visit, parity, type of pregnancy, EIBF professional support, infant sex, colostrum feeding status and family support had such a significant impact on early breastfeeding [4, 16–25].

By recognizing the unquestionable role of the EIBF in reducing infant mortality, the Ethiopian Ministry of Health was targeting to increase the proportion of newborn babies breastfeeding to 92% by 2015 in the first hour of life [26]; however, the Ethiopian Demographic and Health Survey (EDHS) showed that the proportion of children who were breastfed in the first hour of life was 73% and the EIBF region of Amhara was 66% [27].

Although evidence on the prevalence and associated factors of EIBF in different parts of the world, there has been a lack of information on the proportion and associated factors of early breastfeeding among cesarean delivered mothers to date. Therefore, this study aimed to assess the proportion of EIBF among cesarean delivered mothers and to identify the factors affecting EIBF in South Gondar Zone Hospitals, North West Ethiopia, 2020.

## Methods and materials

### Study area and period

The study was conducted in South Gondar Zone Hospitals from 12 June 2020 to 03 July 2020. South Gondar Zone, which is located in the central part of the region of Amhara and the north-western part of Ethiopia. The area is situated about 668 km away from the capital city of Ethiopia, Addis Ababa, and 103 km away from the Bahir Dar city of Amhara. Debre Tabor is the administrative town of the South Gondar Zone. The area has 18 Woredas with a population of 2,609,823 (1,304,911 females and 1,304,912 males). The area also includes eight government hospitals, 96 public health centers, 140 private clinics, and 403 health centers [28].

### Study design

An institutional-based cross-sectional study was conducted.

### Population

The source population was all mothers who delivered by cesarean section in South Gondar Zone hospitals; while all mothers who delivered by cesarean section in South Gondar Zone hospitals during the study period were considered as the study population.

### Eligibility criteria

All mothers who gave birth and registered in the delivery registration book in South Gondar Zone hospitals were included in the study. Whereas mothers delivered under general anesthesia and baby have any health problem which requires separation from the mother; which needs admission to NICU were excluded from the study.

### Sample size determination

The sample size was calculated using the single population proportion formula and the required sample size for this study was determined using the following assumptions; desired precision (d) = 5%, Confidence level = 95% (Zα/2 = ±1.96 value), and the prevalence of early initiation of breastfeeding was 66% [27]. Hence, the final calculated sample size with a 5% non-response rate was 356.

### Sampling procedures

All hospitals that provide a cesarean section were taken to get a sufficient sample. Then, a sample from each hospital was determined using proportional allocation to size (PAS). Finally, simple random sampling was used to select all mothers who delivered by cesarean section to got the desired sample size (see Fig. 1).

**Fig. 1:** . Schematic presentation of sampling procedures in selecting CD mothers in South Gondar zone hospitals, 2020. NB: DGH- Debre Tabor General Hospital, NMH- Nifas Mewucha Hospital, MEH- M/eyesus Hospital, AZHA/Zemen Hospital, EBH- Ebenat Hospital, AGH- Arba Gebeya Hospital, SH- Simada Hospital and AH- Andabet Hospital.

### Study variables

#### Dependent variables

Early initiation of breastfeeding (yes/no)

#### Independent variables

Maternal and husband socio-demographic factors (age, religion, marital status, residence, educational status, occupation); Maternal knowledge on EIBF and breastfeeding experience; Obstetric & health service-related factors (history of ANC visit, place of ANC, number of ANC visits, parity, counseling on EIBF during ANC, professional guidance to initiate BF, type of pregnancy and duration of labor pain) and Social related factors (social/family support on EIBF).

### Operational definitions

#### Early initiation of breast feeding

Mothers who had initiated breastfeeding within one hour after birth [28].

#### Knowledge about early initiation of breast feeding

Mothers were asked eight knowledge related questions regarding EIBF and each correct answer was given a value of 1 and an incorrect answer a value of 0. After computing the sum for each respondent and mean, it was dichotomized into good knowledge ≥ mean, poor knowledge < mean [29].

#### Professional guidance to initiate BF

Professionals, who counsel and assist the mother by showing how to hold the baby, how to practice positioning and attachment to initiate breast feeding within one hour.

#### Social/family support to EIBF

Any attendant who encourages, assist the mother and share experience for the mother to initiate breast feeding within one hour.

### Data collection procedures

#### Instrument

A pretested and structured questionnaire was used for data collection. The questionnaire was adopted after reviewing similar work in professional literature. The tool first prepared in English then translated to Amharic and back to English by a language expert to maintain the consistency of the instrument.

#### Data collector’s selection and training

Eight diploma holder nurses conducted the face to face interviews and four BSc degree midwives supervised the data collection process. The data collectors and supervisors were trained for 1 day about the contents of the questionnaire, methods of data collection, and the aim of the study.

#### Data collection

The study participants were given an introduction about the study as well as the opportunity to ask questions about the study and questionnaires were disseminated.

#### Data quality management

The data collectors were trained for one day about the contents of the questionnaire, methods of data collection, and the aim of the study. Any error, ambiguity, or incompleteness identified was corrected immediately. A pre-test was conducted on 36 mothers who gave birth by cesarean section in Felege Hiwot referral hospital; then the instrument was amended accordingly. The data collection process was supervised by the supervisor and the investigator throughout the data collection period.

#### Data processing, analysis, interpretation and presentation

Once all necessary data obtained, data were checked for completeness. The collected data were entered and cleaned using Epi data version 4.2, then exported to SPSS version 23 for analysis. Descriptive analysis was conducted to summarize the data and the final result of the study was interpreted in the form of text and tables. Binary logistic regression analysis was executed to see the association between independent and dependent variables. All explanatory variables with *p* < 0.2 in bivariable logistic regression were entered into multivariable logistic regression analysis and significant association was identified based on *p* < 0.05 and odds ratio with 95% CI in multivariable logistic regression.

## Result

### Socio-demographic characteristics of the participants

Among the total of 356 mothers, 349 mothers were participated in the study making a response rate of 98.03%. The highest proportion, 138(39.5%) mothers were in the age group of 25–29 years. The mean age of the mother was 26.85 (SD ± 5.26) years. More than three fourth 268(76.8%) of mothers were urban residence. Almost all mothers, 341 (97.7%) were Amhara in ethnicity and 261(74.8%) mothers were Orthodox Christian followers. Regarding the educational status of mothers, 196(56.3%) mothers were completed at least secondary school. Concerning the educational status of the husbands, 244(69.9%) husbands of mothers were attending at least secondary school (see Table 1).

**Table 1:** Socio-demographic characteristics of mothers and their husbands in south Gondar zone hospitals, Northwest, Ethiopia, 2020.

Variable	EIBF(*n*=349)			
	Yes		No	
	Frequency	Percent	Frequency	Percent
Maternal age				
15-19	5	1.4	18	5.2
20-24	47	13.5	48	13.8
25-29	80	22.9	58	16.5
30-34	40	11.5	32	9.2
35 and above	9	2.6	12	3.4
Residence				
Urban	156	44.7	112	32.1
Rural	25	7.2	56	16
Marital status				
Married	175	50.1	150	43
Unmarried^#^	6	1.7	18	5.2
Religion				
Orthodox	134	38.4	127	36.4
Muslim	37	10.6	38	10.9
Others*	10	2.9	3	0.9
Maternal education				
Not formal education	24	6.9	46	13.2
Primary school	47	13.5	48	13.8
Secondary school and above	110	31.5	74	21.2
Husband education				
Not formal education	16	4.6	33	9.5
Primary school	20	4.7	36	10.3
Secondary school and above	145	41.5	99	28.4
Maternal occupation				
Government employed	37	10.6	24	6.9
Self employed	43	12.3	22	6.3
Daily laborer Housewife	5	1.4	15	4.3
Farmer	70	20.1	53	15.2
others	26	7.4	54	15.5
Husband occupation				
Government employed	73	22.5	39	12
Self employed	72	22.2	52	16
Daily laborer	7	2.2	10	3.1
Farmer	23	7.1	48	14.8

Other^*^ protestant, catholic, Jehovah, no religion; ^**#**^ Single, divorced and widowed

### Maternal knowledge on early initiation of breastfeeding and breastfeeding experiences

Two hundred fifty-one (71.9%) of mothers heard about EIBF. Regarding the source of information about EIBF, 314 (90%) of mothers reported that the main source of information about EIBF was health professionals. Almost all mothers, 347 (99.4%) reported that breast milk must be given first for the baby after delivery. Two hundred thirty-one (66.2%) of mothers knew about the recommended time of initiating BF. Concerning maternal knowledge on EIBF, two hundred fifty-one (71.9%) of mothers had good knowledge about EIBF. Regarding BF experience, 179(51.3%) of mothers were experienced in BF (see Table 2).

**Table 2:** Maternal knowledge on EIBF and BF experience in south Gondar zone hospitals, northwest Ethiopia, 2020.

Variable	EIBF & BF(***n***=349)			
	Yes		No	
	Frequency	Percent	Frequency	Percent
Did you hear about BF?				
Yes	189	54.2	62	17.7
No	35	10.02	63	18.05
Source of Information				
Health professional’s	172	49.3	142	40.7
Media	21	6.02	14	4.01
Did you know recommended timing of initiating of BF?				
Yes	178	51	53	15.2
No	21	19.2	51	14.6
Maternal knowledge on EIBF & BF				
Good	227	65.04	24	6.9
Poor	77	22.1	21	6.01
Breast feeding experiences				
Yes	144	14.3	35	10.02
No	120	34.4	50	14.3

### Obstetric and health service-related characteristics of the respondents

Regarding the type of pregnancy, 264 (75.6%) of mothers reported that their pregnancies were intended. Almost all mothers 346 (99.1%) of mothers had a history of ANC visits during their pregnancy. Seventy-two (19.8%) of mothers had got EIBF counseling during ANC visit. Concerning professional guidance to EIBF, two hundred ninety-seven (85.1%) of mothers had professional guidance to EIBF. One hundred eighty-four (52.7%) of mothers were multigravida. Regarding the duration of labor pain, 322 (92.3%) of mothers’ labor pain was less than 12 h (see Table 3).

**Table 3:** Obstetric and health service-related characteristics of mothers versus EIBF among cesarean section mothers in south Gondar zone hospitals, Northwest Ethiopia, 2020.

Variable	EIBF & BF(***n***=349)			
	Yes		No	
	Frequency	Percent	Frequency	Percent
Type of pregnancy				
Intended	161	46.1	103	29.5
Unintended	120	5.7	65	18.6
Place of ANC follow up				
Public institution	71	20.5	137	39.6
Private clinic	63	18.2	18	5.2
NGO maternity center	47	13.6	10	2.9
Number of ANC visit				
Less than four visits	51	14.7	21	6.1
Four and above visits	130	37.6	144	41.6
EIBF counseling during ANC visits				
Yes	227	65.04	24	6.9
No	77	22.1	21	6.01
Duration of labor				
Less than 12 hours	172	49.3	150	43
Greater than 12 hours	9	2.6	18	5.2
Received professional Guidance for EIBF				
Yes	169	48.4	128	36.7
No	12	3.4	40	11.5
Parity				
Primi	66	18.9	99	28.4
Multi	115	33	69	19.8

### Prevalence of early initiation of breastfeeding among mothers delivered by cesarean section

The prevalence of early initiation of breastfeeding among mothers who delivered by cesarean section in South Gondar Zone hospitals were 51.9% with 95% CI (47, 57%).

### Reasons for late initiation of breast feeding

The main reasons for delayed initiation of breastfeeding claimed by the study participants were 58% of cesarean surgery-related pain and discomfort, 34.6% of delayed milk secretion, and 2.8% of late shifting from the recovery room.

### Factors associated with EIBF among mothers delivered by cesarean section

On multivariable logistic regression analysis: Factors such as professional guidance to early initiation breastfeeding, type of pregnancy, number of ANC visits, and breastfeeding experience were significantly associated with EIBF among mothers who delivered by cesarean section. Mothers who had received professional guidance to EIBF were 2.68 times (AOR = 2.68, 95% CI = 1.18, 6.10) more likely to initiate breastfeeding early as compared to those mothers who had not received professional guidance to early initiation of breastfeeding. Mothers who had intended pregnancy were 2.69 times (AOR = 2.69, 95% CI = 1.34, 5.38) more likely to initiate BF early as compared to their counterparts. Mothers who had four and above ANC visits were 2.20 times (AOR = 2.20, 95% CI = 1.24, 3.91) more likely to initiate BF early as compared to those mothers who had less than four ANC visit. Mothers who had breastfeeding experience were 2.25 times (AOR = 2.25, 95% CI = 1.33, 3.75) more likely to initiate breastfeeding within one hour as compared to their counterparts (see Table 4).

**Table 4:** Multivariable analysis of EIBF among mothers who delivered by cesarean section in south Gondar zone hospitals, Northwest, Ethiopia, 2020(*n*= 349).

Variable	EIBF		COR, 95%CI	AOR, 95%CI	***P*** value
	Yes	No			
Residence					
Urban	156	112	3.12 (1.83, 5.30)	1.57 (0.56, 4.39)	0.38
Rural	25	56	1	1	
Maternal education					
No formal education	24	46	1	1	
Primary school	47	48	1.87 (0.99, 3.54)	0.81 (0.32, 2.07)	0.67
Secondary & above	110	74	2.84 (1.60, 5.06)	0.45 (0.16, 1.28)	0.14
Received professional guidance to EIBF					
Yes	169	128	4.40 (2.21, 8.72)	**2.68 (1.18, 6.10)**	0.019^*^
No	12	40	1	1	
No of ANC visit					
> Four	139	79	3.72 (2.35, 5.90)	**2.20 (1.24, 3.91)**	0.007*
≤ Four	42	89	1	1	
Duration of labour					
≤ 12 hours	172	150	2.29 (1.1, 5.25)	1.57 (0.56, 4.40)	0.38
> 12 hours	9	18	1	1	
Type of pregnancy					
Intended	161	103	5.08 (2.90, 8.88)	**2.69 (1.34, 5.38)**	0.005*
Unintended	20	65	1	1	
Knowledge on EIBF					
Good	140	111	1.75 (1.09, 2.81)	1.47 (0.83, 2.61)	0.17
Poor	41	57	1	1	
BF experience					
Yes	111	68	2.33 (1.51, 3.58)	**2.25 (1.35, 3.75)**	0.002*
No	70	100	1	1	

*p- value <0.05, ** p-value <0.01

## Discussion

The study was aimed to determine the prevalence of early initiation of breastfeeding and associated factors among mothers who delivered by cesarean section in South Gondar Zone hospitals in Northwest Ethiopia.

This study revealed that the prevalence of early initiation of breastfeeding within one hour among mothers who delivered by cesarean section was found to be 51.9%. This is lower than the study conducted in different parts of Ethiopia [22, 27, 30]. The variation might be due to differences in the study setting, study population, and time period of the study.

This level of early initiation of breastfeeding was found to be high as compared to the studies done in Bangladesh [31], India [32], Kenya [33], and Egypt [34]. The possible reason for this variation might be variation in the study period, sample size, maternal socio-demographic characteristics like access to information, educational status, the cross-cultural difference in breastfeeding practice, and health service utilization characteristics.

Received professional guidance for early initiation of breastfeeding, the number of antenatal care visits, types of pregnancy, and previous breast-feeding experience were significantly associated with the practice of early initiation of breastfeeding among mothers who delivered by cesarean section.

Mothers who were received professional guidance for early initiation of breastfeeding were 2.68 times more likely to initiate breastfeeding early [AOR = 2.68, 95% CI = (1.18–6.10)] as compared to their counterparts. This finding was supported by a study conducted in Brazil [35], Indonesia [16], Bangladesh [17], and Uganda [18]; which showed that professional assistance or guidance after delivery increase early initiation of breastfeeding by mothers.

This might be because encouragement and motivation from health workers help mothers to take a stand in EIBF practice. A skilled and properly trained health care provider can motivate mothers to initiate early breastfeeding and explain its advantages, counsel on dangers of pre-lacteal feeding and its long-term risk, and the benefits of EIBF and continuation of breastfeeding [36].

ANC frequency was another factor that was significantly associated with EIBF among CD mothers. Those cesareans delivered mothers who had four and above ANC visits were two times more likely to initiate breastfeeding early [AOR = 2.20, 95% CI = (1.24–3.91)] as compared to those who had less than four ANC visit. This finding was consistent with a study conducted in Dembecha [37] and western Ethiopia [20]. This could be because mothers who had frequent antenatal care visits during their pregnancy could access frequent counseling sessions on the importance of EIBF, and thereby more likely to practice it. But the finding of this study was inconsistent with a study conducted in Axum [38] and Debre Birhan [24] which showed that number of ANC visit did not influence EIBF.

Type of pregnancy was also significantly associated with early initiation of breastfeeding among mothers who delivered by cesarean section. According to this finding mothers with intended pregnancy were more likely to initiate BF early [AOR = 2.69, 95% CI = (1.34–5.38)] as compared to mothers with unintended pregnancy which was consistent with a study conducted in Turkey [25] and Nigeria [21]. This could be explained by the fact that a woman’s attitude toward her baby can affect her likelihood of baby-care and consequently her decision to initiate breastfeeding.

Mothers who had previous breastfeeding experience were 2.25 times more likely to initiate breastfeeding within one hour [AOR = 2.25, 95% CI = (1.35–3.75)] as compared to their counterparts. This finding was supported by studies conducted in Tabriz, state of eastern Azerbaijan [19] and Egypt [39]. The reason for this might be due to mothers whose breastfeeding experience might have exposure to professional counseling, their experience on how to breastfeed the baby and experience how to position, and attach the baby might help the mothers to initiate breastfeeding early.

The limitations of this study include; the cross-sectional nature of this study limits to set a causal-effect relationship between dependent and independent variables. Since it is based on mothers report the exact time that is the first one hour after birth might be difficult to measure. Selection bias might be also the limitation of the study.

## Conclusions

The prevalence of early initiation of breastfeeding in the study area was high. Professional guidance to EIBF, type pregnancy, previous breastfeeding experience, and the number of ANC visits were significantly associated with early initiation of breastfeeding among mothers who delivered by cesarean section.

### Recommendations

#### Woreda and Zonal health office

Should focus on strengthening the provision of information, education, and communication family planning methods.

#### Health professionals

Better to provide counseling, health education, and creating awareness of the importance of ANC services as well as timing, techniques, and benefits of breastfeeding.

#### Researchers

Further studies should focus on the qualitative approach to come up with additional findings.

## Data Availability

The datasets used and/or analyzed during the current study are available from the corresponding author on reasonable request.

## Abbreviations

ANC: Antenatal Care
BF: Breast Feeding
CD: Cesarean Delivery
DIBF: Delay Initiation of Breastfeeding
EDHS: Ethiopian Demographic and Health Survey
EIBF: Early Initiation of breastfeeding
NICU: Neonatal Intensive Care Unit
UNICEF: United Nation Children Fund
